# Passive Immunization Reduces Behavioral and Neuropathological Deficits in an Alpha-Synuclein Transgenic Model of Lewy Body Disease

This article has been retracted.

**DOI:** 10.1371/journal.pone.0019338

**Published:** 2011-04-29

**Authors:** Eliezer Masliah, Edward Rockenstein, Michael Mante, Leslie Crews, Brian Spencer, Anthony Adame, Christina Patrick, Margarita Trejo, Kiren Ubhi, Troy T. Rohn, Sarah Mueller-Steiner, Peter Seubert, Robin Barbour, Lisa McConlogue, Manuel Buttini, Dora Games, Dale Schenk

**Affiliations:** 1 Department of Neurosciences, University of California San Diego, La Jolla, California, United States of America; 2 Department of Pathology, University of California San Diego, La Jolla, California, United States of America; 3 Department of Biology, Boise State University, Boise, Idaho, United States of America; 4 ELAN Pharmaceuticals, South San Francisco, California, United States of America; The University of Hong Kong, Hong Kong

## Abstract

Dementia with Lewy bodies (DLB) and Parkinson's Disease (PD) are common causes of motor and cognitive deficits and are associated with the abnormal accumulation of alpha-synuclein (α-syn). This study investigated whether passive immunization with a novel monoclonal α-syn antibody (9E4) against the C-terminus (CT) of α-syn was able to cross into the CNS and ameliorate the deficits associated with α-syn accumulation. In this study we demonstrate that 9E4 was effective at reducing behavioral deficits in the water maze, moreover, immunization with 9E4 reduced the accumulation of calpain-cleaved α-syn in axons and synapses and the associated neurodegenerative deficits. In vivo studies demonstrated that 9E4 traffics into the CNS, binds to cells that display α-syn accumulation and promotes α-syn clearance via the lysosomal pathway. These results suggest that passive immunization with monoclonal antibodies against the CT of α-syn may be of therapeutic relevance in patients with PD and DLB.

## Introduction

Neurodegenerative conditions with accumulation of α-synuclein (α-syn) are common causes of dementia and movement disorders in the aging population. Disorders where the clinical and pathological features of Alzheimer's Disease (AD) and Parkinson's Disease (PD) overlap are known as Lewy body disease (LBD) [1].

α-Syn is a natively unfolded protein [2] found at the presynaptic terminal [3] and may play a role in synaptic plasticity [4]. Abnormal α-syn accumulation in synaptic terminals and axons plays an important role in LBD [5], [6], [7], [8]. Recent work has suggested that α-syn oligomers rather than fibrils might be the neurotoxic species [9], [10].

While in rare familial cases mutations in α-syn might contribute to oligomerization [11], it is unclear what triggers α-syn aggregation in sporadic forms of LBD. Alterations in α-syn synthesis, aggregation or clearance have been proposed to impact the formation of toxic oligomers [12], [13], [14]. Therefore, strategies directed at promoting the clearance of oligomers may be of therapeutic value for LBD. Previous studies have used gene therapy targeting selective regions to increase α-syn clearance via autophagy or by reducing α-syn synthesis [12], [15].

However, neurodegenerative processes in LBD are more widespread than originally suspected [16] therefore there is a need for therapeutic approaches that target toxic α-syn in multiple neuronal populations simultaneously. For this reason we began to explore an immunotherapy approach for LBD and have previously shown that active immunization with recombinant α-syn ameliorates α-syn related synaptic pathology in a transgenic (tg) mouse model of PD [17]. Previous studies have shown that intracellular antibodies (intrabodies) can inhibit α-syn aggregation [18], [19] and that copolymer-1 immunotherapy reduces neurodegeneration in a PD model [20].

The mechanisms through which α-syn immunotherapy might work are unclear given that native α-syn is cytoplasmic. However, it is possible that antibodies may recognize abnormal α-syn accumulating in the neuronal plasma membrane [10], [17], [21], [22] or secreted forms of α-syn. In support of this possibility, studies have shown that oligomerized α-syn is secreted in vitro [23] and in vivo [24] via exocytosis, contributing to the propagation of the synucleinopathy. Moreover, α-syn is present in the cerebrospinal fluid of α-syn tg mice and in patients with LBD [25], [26].

This study examined whether passive immunization with an antibody against the C-terminus (CT) of α-syn (hereafter referred to as the 9E4 antibody) was able to recognize and clear a-syn aggregates in a-syn tg mice. We show that the 9E4 antibody crossed into the CNS and ameliorated behavioral deficits and neuropathological alterations in α-syn transgenic mice. In addition we show that 9E4 is able to reduce the accumulation of calpain-cleaved and oligomerized a-syn aggregates. These results imply that passive immunization against the CT of α-syn may be an important therapeutic alternative in patients with PD and DLB.

## Materials and Methods

### Transgenic mouse model and passive immunization

For this study mice over-expressing α-syn under the PDGF-β promoter (Line D) were utilized [27], [28]. This model was selected because mice from this line develop α-syn aggregates distributed through the temporal cortex and hippocampus similar to what has been described in LBD accompanied by behavioral deficits [29], [30].

Initial immunoblot and immunohistochemical studies were conducted with a panel of antibodies directed at both N-terminus (NT) (6H7) and CT-α-syn (8A5, 9E4) to determine which of these antibodies displayed the most specific binding to human α-syn, of these antibodies, 9E4 displayed the most specificity and was chosen for the immunization study. A total of 40 α-syn tg mice (6 m/o, n = 20 mice per group) received weekly intraperitoneal (IP) injections (10 mg/kg) for 6 months with the CT-α-syn antibody (9E4) and IgG1 control. An additional group of non-tg mice treated with the 9E4 antibody (n = 12) and the IgG1 control (n = 12) was included as control for behavioral and neuropathological studies. Mice were bled once a month and antibody titers monitored by enzyme-linked immunosorbent assay (ELISA). At the end of the studies, mice were tested for functional effects in the water maze. Brains and peripheral tissues were removed and divided sagittally.

For studies of antibody trafficking into the CNS the mouse monoclonal antibody 9E4 was concentrated with a 10-kDa cutoff concentrator centrifuge tube (Millipore, Temecula, CA) and linked to the Fluorescein isothiocyanate (FITC) molecule utilizing a FluoroTag FITC conjugation kit (Sigma-Aldrich, St. Louis, MO) according to the manufacturer's instructions. For this experiment non-tg (total n = 18) and α-syn tg mice (total n = 18) (6 m/o) were injected intravenously (IV) with the 9E4-FITC or a non-immune control FITC tagged IgG1 at a concentration of 1 mg/kg. Mice were sacrificed 3, 14 and 30 days after injection (n = 3 per group). CSF from these mice was used to immunolabel cortical sections from antibody-naive animals.

As an additional control to monitor the passage of FITC-labeled antibodies across the blood-brain barrier, mice were injected with FITC tagged **β**-syn. The For this experiment non-tg (total n = 8) and α-syn tg mice (total n = 8) (6 m/o) were injected intravenously (IV) with the FITC-labeled β-syn or a non-immune control FITC tagged IgG1 at a concentration of 1 mg/kg. Mice were sacrified at 14 days post-injection. CSF from these mice was also used to immunolabel slides from FITC tagged **β**-syn niave non-tg and α-syn tg mice.

Upon sacrifice, the right hemibrain was post-fixed in phosphate-buffered 4% PFA (pH 7.4) at 4°C for 48 hours for neuropathological analysis, while the left hemibrain was snap-frozen and stored at −70°C for subsequent protein analysis. All experiments described were approved by the animal subjects committee at the University of California at San Diego (UCSD) and were performed according to NIH recommendations for animal use. UCSD is an Institutional Animal Care and Use Committee accredited institution and the UCSD Animal Subjects Committee approved the experimental protocol (S02221) followed in all studies according to the Association for Assessment and Accreditation of Laboratory Animal Care International guidelines.

### Preparation of antibodies for passive immunization

Previous active immunization experiments have suggested that the most effective antibodies were against CT-epitopes of α-syn [17], for this study a panel of antibodies were developed 1) clone 8A5 (α-syn epitope 125–140; IgG1); 2) clone 9E4 (α-syn epitope 118–126; IgG1) and 6H7 (α-syn epitope 1–4: IgG1) (Table 1). The 9E4 and 6H7 antibodies were prepared by immunizing with recombinant human α-syn, while 8A5 was generated with purified bovine α-syn. Epitope mapping was done on 15-mer peptides that had a 3 amino acid difference (i.e. 1–15, 3–18, etc, which gave an epitope resolution of +/−2 amino acids). For control experiments a non-immune IgG1 (clone 27-1) prepared under similar conditions was used. Initial immunoblot and immunohistochemical examination using these antibodies on untreated non-tg and α-syn tg mice demonstrated that the 9E4 displayed the most specificity for human α-syn therefore this antibody was chosen for the immunization study.

**Table 1:** Antibodies used for this study.

Antibodyname	Type of antibody	Epitope/specificity	Antibody Isotype	ExperimentalUse
27-1	Monoclonal	Control	IgG1	Control for Immunization
6H7	Monoclonal	NT 1-4	IgG1	Initial Characterization
8A5	Monoclonal	CT 125-140	IgG1	InitialCharacterization
9E4	Monoclonal	CT 118-126	IgG1	Passive Immunization
FL-α-syn	Polyclonal	FL	Affinity purified	ICC and IB
CC-α-syn	Polyclonal	CT 122-123	Affinity purified	ICC and IB

CT =  C-terminus; FL =  full length; CC  =  Calpain-cleaved; ICC =  immunocytochemistry; IB =  Immunoblot.

### Behavioral testing

#### Water maze

In patients with LBD, α-syn accumulates not only in subcortical nuclei but also in the temporal cortex and limbic system and accounts for cognitive deficits in these patients [31]. Similarly, in our PDGF-α-syn tg mice, protein accumulation occurs in the temporal cortex and hippocampus [28]. In this context and as previously described [29], in order to evaluate the functional effects of passive immunization treatment in mice, groups of non-tg and α-syn tg animals were tested in the water maze. For this purpose, a pool (diameter 180 cm) was filled with opaque water (24°C) and mice were first trained to locate a visible platform (days 1–3) and then a submerged hidden platform (days 4–7) in three daily trials 2–3 min apart. Mice that failed to find the hidden platform within 90 seconds were placed on it for 30 seconds. The same platform location was used for all sessions and all mice. The starting point at which each mouse was placed into the water was changed randomly between two alternative entry points located at a similar distance from the platform. In addition, on the final day of testing the platform was removed and the time spent by mice in the correct quadrant was measured (Probe test). The duration of the probe test was 40 secs. Time to reach the platform (escape latency) was recorded with a Noldus Instruments EthoVision video tracking system (San Diego Instruments, San Diego, CA) set to analyze two samples per second.

#### Pole Test

For the pole test, animals were placed head upward on top of a vertical wooden pole 50 cm long and 1 cm in diameter. When placed on the pole, animals orient themselves downward and descend the length of the pole. Groups of mice received training that consisted of five trials for each session. For testing, animals received five trials and the time taken to descend (T-total) was measured.

#### Rotarod

Mice were analyzed for 2 days in the Rotarod (San Diego Instruments, San Diego, CA), as previously described (Masliah et al., 2000). On the first day, mice were trained for five trials: the first one at 10 rpm, the second at 20 rpm, and the third to the fifth at 40 rpm. On the second day, mice were tested for seven trials at 40 rpm each. Mice were placed individually on the cylinder and the speed of rotation increased from 0 to 40 rpm over a period of 240 s. The length of time mice remained on the rod (fall latency) was recorded and used as a measure of motor function.

### ELISA analysis of brain and plasma antibody concentrations

Antibody levels in the brain and plasma of immunized mice were determined as previously described [17]. Briefly, using 96-well microtiter plates coated with 0.4 µg per well of purified full-length α-syn. Samples were incubated overnight followed by goat anti-mouse IgG alkaline phosphatase-conjugated antibody (1∶7500, Promega, Madison, WI). The plate was read at wavelengths of 450 nm and 550 nm. Results were plotted on a semi-log graph with relative fluorescence units versus serum dilution. Antibody titer was defined as the dilution at which there was a 50% reduction from the maximal antibody binding.

### Immunoblot analysis

Briefly, as previously described, brains were homogenized and divided into cytosolic and membrane fractions [12], [15]. For immunoblot analysis, 20 µg of total protein per lane was loaded into 4–12% Bis-Tris SDS-PAGE gels and blotted onto polyvinylidene fluoride (PVDF) membranes. For characterization of the antibodies samples from untreated non-tg and α-syn tg mice were incubated the with monoclonal antibodies against CT and N-Terminal (NT) α-syn (9E4, 6H7 and 8A5, ELAN Pharmaceuticals). To determine the effects of the immunotherapy in levels of α-syn blotted samples from treated α-syn tg were probed with antibodies against calpain-cleaved α-syn (CC α-syn) which recognizes a C-terminal fragment of α-syn [32], full length α-syn (FL α-syn rabbit polyclonal (1∶1000, Millipore, Temecula CA). For the analysis of synaptic proteins, monoclonal antibodies against Synapsin I (1∶1000, Millipore, Temecula, CA) and PSD95 (UC Davis/NIH Neuro-Monoclonal Antibody Facility, Davis, CA) were used. In order to determine the effects of the immunotherapy on levels of total tau and PHF-tau blotted samples from treated α-syn tg were probed with antibodies against total tau (1∶1000, Dako, Carpinteria, CA) and PHF-tau (1∶1000, UC Davis/NIH Neuro-Monoclonal Antibody Facility, Davis, CA). Incubation with primary antibodies was followed by species-appropriate incubation with secondary antibodies tagged with horseradish peroxidase (1∶5000, Santa Cruz Biotechnology, Santa Cruz, CA), visualization with enhanced chemiluminescence and analysis with a Versadoc XL imaging apparatus (BioRad, Hercules, CA). Analysis of β-actin (Sigma) levels was used as a loading control.

### Immunocytochemical and neuropathological analyses

For characterization of the antibodies used for immunotherapy, vibratome sections from untreated non-tg and α-syn tg mice were incubated the with monoclonal antibodies against CT and NT-α-syn (9E4, 6H7 and 8A5, ELAN Pharmaceuticals). Analysis of α-syn accumulation for the immunotherapy experiment was performed in serially-sectioned, free-floating, blind-coded vibratome sections by incubating the sections overnight at 4°C with a polyclonal antibody against total α-syn (1∶500, affinity purified rabbit polyclonal, Millipore) [27] and with an antibody against the calpain-cleaved CT-α-syn [32], followed by secondary antibodies tagged with FITC or biotinylated goat anti-rabbit IgG1 (1∶100, Vector Laboratories, Inc., Burlingame, CA), Avidin D-HRP (1∶200, ABC Elite, Vector) and detection with the Tyramide Signal Amplification™-Direct (Red) system (1∶100, NEN Life Sciences, Boston, MA). In order to determine the effects of immunotherapy on levels of total tau and PHF-tau blotted samples from treated α-syn tg were probed with antibodies against total tau (1∶500, Dako, Carpinteria, CA) and PHF-tau (1∶500, UC Davis/NIH Neuro-Monoclonal Antibody Facility, Davis, CA). Antibodies against Zo-1 (1∶500, Millipore, Temecula, CA), Iba-1 (1∶1000, Wako, Richmond, VA) and GFAP (1∶1000, Millipore, Temecula, CA) were used to examine the effects of passive immunization with 9E4 on vasculature or glial cell activation respectively. All sections were processed simultaneously under the same conditions and experiments were performed in triplicate in order to assess the reproducibility of results.

Stereological analysis and quantification of neocortical and hippocampal intra-neuronal FL-αsyn and CC-αsyn immunoreactivity was conducted by the disector method using the Stereo-Investigator System (MBF Bioscience, Williston, VT) and the results were averaged and expressed as cell counts per 0.1 mm^3^. Neocortical and hippocampal FL-αsyn and CC-αsyn immunoreactive neuropil was assessed in digital images analyzed with the Image Quant software by selecting and area to exclude cell bodies, setting the threshold levels and expressing the data as pixel intensity (arbitary units).

### Double immunolabeling and fluorescence co-labeling

To determine the co-localization between α-syn and lysosomal and autophagy markers double-labeling experiments were performed, as previously described [15]. For this purpose, vibratome sections were immunolabeled with the rabbit polyclonal antibodies against α-syn (Millipore, affinity purified polyclonal, 1∶500) or CC α-syn [27], [32] and LC3 (Abcam) or cathepsin-D (Dako, 1∶100). The α-syn immunoreactive structures were detected with the Tyramide Signal Amplification™-Direct (Red) system (1∶100, NEN Life Sciences, Boston, MA) while LC3 and cathepsin-D was detected with FITC tagged antibodies (Vector, 1∶75). Co-labeling experiments were performed with antibodies against cathepsin-D and LC3 detected with tyramide red in sections from mice that received IV injections with the 9E4-FITC or IgG1-FITC. All sections were processed simultaneously under the same conditions and experiments were performed in triplicate in order to assess the reproducibility of results. Sections were imaged with a Zeiss 63X (N.A. 1.4) objective on an Axiovert 35 microscope (Zeiss) with an attached MRC1024 LSCM (laser scanning confocal microscope) system (BioRad) [27].

### Electron microscopy and immunogold analysis

Briefly, vibratome sections were postfixed in 1% glutaraldehyde, treated with osmium tetraoxide, embedded in epon araldite and sectioned with the ultramicrotome (Leica, Germany). Grids were analyzed with a Zeiss OM 10 electron microscope as previously described [33]. For immunogold labeling, sections were mounted in nickel grids, etched and incubated with biotin-tagged antibodies against mouse IgG1 to detect the circulating antibodies utilized for immunization or with antibodies against α-syn followed by labeling with 10 nm Aurion ImmunoGold particles (1∶50, Electron Microscopy Sciences, Fort Washington, PA) with silver enhancement. A total of 125 cells were analyzed per condition. Cells were randomly acquired from 3 grids, and electron micrographs were obtained at a magnification of 25,000X.

For morphometric analysis of synapses from each section, a total of 20 electron micrographs were obtained at a final magnification of 12,000x. Electron micrographs were digitized and analyzed with the Quantimet 570C (Leica, Deerfield, IL) to determine the density of synapses per unit of volume.

### Neuronal cell cultures and treatments

The rat neuroblastoma cell line B103 was used for *in vitro* experiments [34]. This model was selected because over expression of α-syn in these cells interferes with neuronal plasticity (reduced neurite outgrowth and adhesion) but does not result in overt cell death [35], [36]. This model mimics the early pathogenic process of PD where cell death is preceded by reduced neurite outgrowth and synaptic alterations. For all experiments, cells were plated in complete media (Dulbecco's Modified Eagle Medium [Invitrogen, Carlsbad, CA] supplemented with 10% fetal bovine serum (Irvine Scientific, Santa Ana, CA) and infected with LV expressing α-syn or controls at a multiplicity of infection (MOI) of 40. After infection, cells were incubated for 48 hr in a humidified 5% CO_2_ atmosphere at 37°C. All experiments were conducted in triplicate to ensure reproducibility. To investigate the effects of the antibody treatment on autophagy and α-syn, neuronal cells were grown as described above and were then plated onto poly L-lysine coated glass coverslips at a density of 5×10^4^ cells. Five hours after plating, cells were infected with the LV-αsyn LV-control and incubated for 24 hours with 9E4 (3 µg/ml) or IgG1 control in the presence or absence of inhibitors of the autophagy pathway – 3-methyladenine (3-MA, 10 mM, Sigma) or inducers – rapamycin (200 nM, Sigma) as previously described [15]. All coverslips were also co-infected with an LV expressing LC3-GFP at an MOI of 40. Cultures were then washed 2X with serum-free DMEM and then fed either complete media or serum-free media for 12 hours before fixation with 4% PFA. Briefly as previously described [37], coverslips were treated with Prolong Gold anti-fading reagent with DAPI (Invitrogen) and imaged with the LSCM to determine the number of GFP-positive granular structures consistent with autophagolysosomes using semiautomatic image analysis system and the ImageQuant software. For each condition an average of 50 cells were analyzed.

### Statistical analysis

All experiments were done blind-coded and in triplicate. Values in the figures are expressed as means ± SEM. To determine the statistical significance, values were compared using one-way analysis of variance (ANOVA) with post hoc Dunnett's test when comparing to the IgG1 control. Additional comparisons were done using Tukey-Kramer or Fisher post hoc tests. Repeated-measures two-way ANOVA was used to analyze the water maze and Rotarod data when comparing immunized mice to the non-tg or IgG1 treated controls. The differences were considered to be significant if p values were less than 0.05.

## Results

### Initial characterization of novel monoclonal α-syn antibodies and selection of antibody for passive immunotherapy in α-syn tg mice

The PDGFβ-α-syn tg mice were selected for the present study as they display accumulation of α-syn in cortical and sub-cortical regions and neuropathological and behavioral deficits consistent with LBD [12], [17], [27], [28], [29], [38]. In order to initially characterize the specificity of the mouse monoclonal antibodies and to select the one to be used for immunotherapy (Table 1) tissue sections and brains homogenates from non-tg and α-syn tg mice were examined by immunoblot and immunohistochemistry.

By immunoblot analysis (Figure S1A), the NT-α-syn antibody (6H7) identified the α-syn monomer at 14 kDa in both the α-syn tg mice and to a lesser degree in the non-tg mice. The antibodies against CT- αsyn (8A5, 9E4) antibodies specifically recognized the α-syn monomer at 14 kDa in the α-syn tg mice (Figure S1A). No immunoreactivity was observed with the IgG1 control (Figure S1A). The FL α-syn antibody recognized monomeric α-syn in the α-syn tg mice (Figure S1A). Consistent with a previous report [32] the antibody against the calpain-cleaved (CC) α-syn, which recognizes a C-terminally cleaved fragment of α-syn, produced a distinctive pattern detecting a native band at 14 kDa. No cross-reactivity was observed with these antibodies in the non-tg animals (Figure S1A).

Immunohistochemical analysis demonstrated that, compared to the non-immune IgG1, (Figure S1B, C) antibodies against the NT (6H7) (Figure S1D,E) and CT of α-syn (8A5) (Figure S1F, G), (9E4) (Figure S1H,I) strongly immunolabeled the neuropil and the intra-neuronal α-syn aggregates in the temporal cortex of the α-syn tg mice. In the non-tg mice, there was a mild immunoreactivity with the 8A5 antibody (Figure S1F), which was more prominent with the 6H7 antibody (Figure S1D). With the 9E4 antibody no immunoreactivity was detected in the non-tg mice (Figure S1H).

The patterns of immunostaining of the antibodies used for immunotherapy were compared to a polyclonal antibody against FL-α-syn (Figure S1J, K) and to the antibody against CC-α-syn, (Figure S1L,M). In the α-syn tg mice, both antibodies immunolabeled the intra-neuronal α-syn aggregates and the neuropil. The polyclonal antibody against FL α-syn immunolabeled the neuropil in the non-tg mice (Figure S1J), no immunoreactivity was detected with the antibody against calpain-cleaved α-syn in these mice (Figure S1L).

Collectively these results demonstrate that the 9E4 antibody directed against the CT of α-syn displayed the most specificity for human α-syn, therefore this antibody was chosen for the subsequent passive immunization study.

### An antibody against CT-α-syn ameliorates motor and learning deficits and synaptic pathology in α-syn tg mice

Following the initial screening and subsequent selection of the 9E4 antibody, α-syn tg and non-tg mice were passively immunized with either 9E4 or the control IgG1. Antibody titers in the passively immunized α-syn tg and non-tg mice were analyzed by ELISA. On average titer levels were comparable between passively immunized α-syn tg and non-tg mice, though a greater variability was observed within the α-syn tg group (Figure 1A).

**Figure 1:** Plasma antibody titers and effects of passive immunization on motor behavior in passively immunized α-syn tg mice. (A) Antibody titers determined by ELISA in non-tg or α-syn tg mice immunized with the C-terminal antibody (9E4) or IgG1 controls. Horizontal lines represent the mean of the data, whilst the points represent the spread of the individuals in each group. To examine the effects of immunization with the 9E4 antibody on motor behavior in the α-syn tg, mice were tested in the rotarod and pole tests. (B) Pole test performance (time taken to traverse pole) by non-tg mice or α-syn tg mice immunized with IgG1 or 9E4. N = 20 mice per group; 12 month old. Error bars represent mean ± SEM. (C) Rotarod performance (time spent on rotating rod) by non-tg mice or α-syn tg mice immunized with IgG1 or 9E4. Error bars represent mean ± SEM. When analyzing rotarod results (*) indicates p<0.05, when comparing α-syn tg immunized with IgG1 to non-tg group by repeated-measures two-way ANOVA and (#) indicates p<0.05, when comparing α-syn tg mice immunized with 9E4 to IgG1 immunized α-syn tg mice using repeated-measures two-way ANOVA. When analyzing pole test results (*) indicates p<0.05, when comparing α-syn tg immunized with IgG1 to non-tg group by one-way ANOVA with post hoc Dunnett's and (#) indicates p<0.05, when comparing α-syn tg immunized with 9E4 to IgG1 immunized α-syn tg mice by one-way ANOVA with post hoc Dunnett's.

The effects of passive immunization on motor behavior in the α-syn tg mice was assessed using the rotarod and pole test. Results from the pole test demonstrated a motor impairment in the IgG1-treated α-syn tg mice compared to IgG1-treated non-tg mice, evidenced by the significantly longer time taken by the α-syn tg mice to traverse the pole as determined by one-way ANOVA (Figure 1B). Immunization with the 9E4 antibody significantly reduced the time taken by the α-syn tg mice to traverse the pole when compared to IgG1-treated α-syn tg mice (Figure 1B). The time taken to traverse the pole by the α-syn tg mice immunized with the 9E4 antibody did not significantly different from the time taken by the non-tg mice, as determined by one-way ANOVA (Figure 1B).

Statistical analysis of the Rotarod results using repeated-measures two-way ANOVA demonstrated that IgG1-treated α-syn tg mice spent significantly less time on the rotating rod in comparison to IgG1-treated non-tg mice, suggesting that the α-syn tg mice have deficits in motor coordination (Figure 1C). In contrast, α-syn tg mice immunized with the 9E4 antibody spent a significantly longer time on the rod when compared to IgG1-treated α-syn tg mice, as determined by repeated-measures two-way ANOVA (Figure 1C). The time spent on the rod by α-syn tg mice immunized with the 9E4 antibody did not differ from that of the non-tg controls.

In order to evaluate the effects of passive immunization with the CT α-syn antibody on memory and learning, following the 6-month immunization period, mice were tested in the water maze. During the initial training part of the test when the platform was visible (days 1-3), all groups performed at comparable levels, though a greater variability was observed in the IgG1-treated α-syn tg mice (Figure 2A, B, cued platform), as determined by repeated measures two-way ANOVA. At day 2 of the visible platform 9E4-treated α-syn tg appear to reach the platform at a faster rate compared to the other 3 group. However at the end of the visible period of training all 4 groups of mice performed similarly. Following the cued platform session, the mice underwent 4 days of testing during which the platform was submerged and hidden from view (days 4–7). On the first day of testing with the hidden platform all groups performed comparably, indicating that that were all able to swim and locate the platform. Over the next 3 days of testing the performance of the non-tg mice improved in terms of the distance of their swim path and the time taken to locate the platform, During the submerged platform segment of the test, the performance of the IgG1-treated α-syn tg mice did not improve to the same extent as that observed in the non-tg mice (Figure 2A, B, hidden platform). Upon statistical analysis of performance with the submerged platform (days 4–7) using repeated-measures two-way ANOVA a significant difference was observed between the IgG1-treated α-syn tg mice and non-tg controls, with the IgG1-treated α-syn mice taking a significantly longer path and longer time to locate the hidden platform in comparison to their non-tg littermates (Figure 2A, B, hidden platform). These results indicate that the α-syn tg mice have a deficit in the learning and memory skills associated with this task.

**Figure 2:** Effects of passive immunization on behavioral performance in the water maze in passively immunized α-syn tg mice. (A) Performance in the water maze (distance taken to locate platform) during training with the cued platform (days 1–3) and with the platform submerged (days 4–7) in non-tg mice or α-syn tg mice immunized with IgG1 or 9E4. (B) Performance in the water maze (time to locate the platform) during training with the cued platform (days 1–3) and with the platform submerged (days 4–7) in non-tg mice or α-syn tg mice immunized with IgG1 or 9E4. (C) Probe test performance (time spent in correct quadrant) (day 8) in non-tg mice or α-syn tg, mice immunized with IgG1 or 9E4. N = 20 mice per group; 12 month old. Error bars represent mean ± SEM. (D) Representative images of the swim paths of animals from each group when the platform was visible (Day 3, trial 4, red box indicates the location of the platform), hidden (Day 7, trial 4, red box indicates the location of the platform which is now submerged below the opaque surface) or absent (Day 8, Probe Test). When analyzing the water maze results (*) indicates p<0.05, when comparing α-syn tg immunized with IgG1 to non-tg IgG1 group by repeated-measures two-way ANOVA and (#) indicates p<0.05, when comparing α-syn tg immunized with 9E4 to IgG1 immunized α-syn tg mice by repeated-measures two-way ANOVA. When analyzing probe test results (*) indicates p<0.05, when comparing α-syn tg immunized with IgG1 to non-tg IgG1 group by one-way ANOVA with post hoc Dunnett's and (#) indicates p<0.05, when comparing α-syn tg immunized with 9E4 to IgG1 immunized α-syn tg mice by one-way ANOVA with post hoc Dunnett's.

Analysis using repeated-measures two-way ANOVA demonstrated that mice immunized with the 9E4 antibody took a significantly shorter path and time to locate the hidden platform in comparison to IgG1-treated α-syn tg mice (Figure 2A, B, hidden platform), indicating that passive immunization with this antibodies was able to ameliorate the memory and learning deficit observed in the IgG1-treated α-syn tg mice. The time taken by the 9E4 immunized α-syn tg mice to find the submerged platform did not differ significantly from that of the non-tg mice as determined by repeated-measures two-way ANOVA. In the non-tg mice immunization with the 9E4 antibody or the IgG1 control had no deleterious effect upon their performance during the cued or hidden portions of the water maze test (Figure 2A, B).

Following the final day of testing with the submerged platform the mice underwent a Probe test. During this test the platform was removed completely and the time spent by the mice in the correct quadrant (that corresponding to the previous location of the platform) was measured. A longer time spent in the correct quadrant is indicative of a learning effect wherein the mice remember the previous location of the platform and spend an increased period of time looking for it, whilst a shorter time in this quadrant indicates a memory deficit. Statistical analysis using one-way ANOVA demonstrated a significant decrease in the amount of time spent in the correct quadrant by IgG1-treated α-syn tg mice in comparison to non-tg control mice (Figure 2C) suggestive of a memory deficit in these mice. In contrast, α-syn tg mice immunized with the 9E4 antibody spent longer in the target area when compared to IgG1-treated α-syn tg mice, as determined by one-way ANOVA (Figure 2C). The time spent in the correct quadrant by α-syn tg mice immunized with the 9E4 antibody did not differ from that of the non-tg controls. These results suggest that immunization with the 9E4 antibody was able to ameliorate the memory deficits observed in the IgG1-treated α-syn tg mice. No significant effects were observed in the probe test in non-tg mice treated with the 9E4 antibody or the IgG1 control (Figure 2C).

Representative images of the swim paths of mice from the different groups are shown in Figure 2D for day 3, trial 4 (platform visible, red box indicates location of platform) and day 7, trial 4 (platform hidden, red box indicates location of platform which now submerged in the opaque water). When the platform was visible all mice appeared to take a comparable path length to the platform (Figure 2A D- Day 3, trial 4, Platform visible). When the platform was submerged, IgG1-treated α-syn tg mice took a significantly longer path and a more convoluted path to find the platform (Figure 2A, D - Day 7, trial 4, Platform hidden). In contrast, 9E4-immunized α-syn tg mice were able to locate the hidden platform with a time comparable to that observed in the IgG1-treated non-tg controls and with a much more direct path than that observed with IgG1-treated α-syn tg mice (Figure 2A, D - Day 7, trial 4, Platform hidden). In the probe test portion of the water maze IgG1-treated α-syn tg mice did not spend a significant amount of time in the correct quadrant (Figure 2C, D - Day 8, Probe Test). In contrast, the α-syn tg mice that had been immunized with 9E4 spent much longer in the correct quadrant, comparable to the time observed in the IgG1-treated non-tg controls (Figure 2C, D - Day 8, Probe Test).

Since improvements in behavioral performance may be related to enhanced synaptic connectivity, synaptic structure was analyzed by electron microscopy. Ultrastructural analysis (Figure 3) showed that, compared to non-tg mice (Figure 3A), α-syn tg mice treated with IgG1 displayed a significant reduction in the number of postsynaptic densities (PSDs) and presynaptic terminal diameter (Figure 3C, E, F), as determined by one-way ANOVA. In contrast, immunization with the 9E4 antibody significantly increased the number of PSDs (Figure 3D, E) and the diameter of pre-synaptic terminals in the immunized α-syn mice (Figure 3D, F) in comparison to the IgG1-treated α-syn tg mice, as determined by one-way ANOVA. PSD number and pre-synaptic terminal diameter in the α-syn tg mice immunized with the 9E4 antibody did not significantly differ from that in the non-tg mice (Figure 3A, D, E, F).

**Figure 3:** Analysis of the effects of passive immunization on synaptic structure and markers in α-syn tg animals. The effect of immunization with the 9E4 antibody on synaptic markers was evaluated in the temporal cortex of non-tg and α-syn tg mice by electron microscopy and immunoblot analysis. Representative electron micrographs are from the temporal cortex layers 5–6 obtained at 15,000 X. (A) non-tg mice immunized with IgG1 control. (B) non-tg mice immunized with 9E4. (C) α-syn tg mice immunized with the IgG control. (D) α-syn tg mice immunized with the 9E4 antibody. (E, F) Image analysis of the numbers of post-synaptic densities (PSD) and mean presynaptic terminal diameters respectively. (G) Representative immunoblot for PSD95, a postsynaptic marker and Synapsin I, a presynaptic marker, in non-tg mice or α-syn tg mice immunized with the IgG control or the 9E4 antibody. (H, I) Analysis of the levels of PSD95 and Synapsin I immunoreactive bands respectively. N = 20 mice per group; 12 month old. Error bars represent mean ± SEM. (*) indicates p<0.05, when comparing IgG1-immunized α-syn tg mice to IgG1-immunized non-tg mice and (#) indicates p<0.05 when comparing α-syn tg mice immunized with 9E4 to IgG1 immunized α-syn tg mice using one-way ANOVA with post hoc Dunnett's.

Consistent with the ultrastructural examination, immunoblot analysis (Figure 3G) demonstrated that levels of PSD95 were significantly reduced in the IgG1 treated α-syn tg mice compared to non-tg mice, as determined by one-way ANOVA (Figure 3G, H). The mice immunized with the 9E4 antibody displayed significantly higher levels of PSD95 when compared to IgG1-treated α-syn tg mice, as determined by one-way ANOVA (Figure 3G, H). PSD levels in mice immunized with the 9E4 antibody were not significantly different from those in non-tg mice, as determined by one-way ANOVA (Figure 3G, H). Similarly, immunoblot analysis of Synapsin I, a presynaptic marker, demonstrated significantly reduced levels in the IgG1 treated α-syn mice in comparison to non-tg control mice (Figure 3G, I). Immunization with the CT-α-syn antibody 9E4 significantly increased synapsin levels in the immunized α-syn tg mice in comparison to the IgG1-treated α-syn tg mice (Figure 3G, I), as determined by one-way ANOVA. Synapsin levels in the 9E4-immunized α-syn tg mice did not differ significantly from those observed in the non-tg mice (Figure 3G, I).

In the non-tg mice immunization with the 9E4 antibody or IgG1 control had no deleterious effects upon PSDs, pre-synaptic terminals or on synapsin I levels (Figure 3A, B, E-I).

### Passive immunotherapy with a CT α-syn antibody reduces the accumulation of calpain-cleaved α-syn aggregates

To investigate whether the behavioral and synaptic improvements in the immunized α-syn tg mice were associated with reduced accumulation of α-syn, immunochemical studies were performed with antibodies against FL and CC α-syn. CC-α-syn has been proposed to serve as a substrate for aggregation and antibodies against this epitope have been shown to identify abnormal α-syn aggregates that otherwise are not detected in control human brain or in wild-type mice [32]. With the polyclonal FL α-syn antibody there was no significant difference in the intra-neuronal inclusions in the temporal cortex in 9E4-treated α-syn tg mice in comparison to IgG1-treated α-syn tg mice (Figure 4C, D, I), however there was a small but significant reduction of α-syn immunoreactivity in the neocortical neuropil of the 9E4 treated mice in comparison to IgG1-treated α-syn tg mice (Figure 4C, D, J). In the hippocampus there were no significant differences in FL α-syn immunoreactivity in intra-neuronal inclusions or neuropil between the 9E4-treated α-syn tg mice and IgG1-treated α-syn tg mice control groups (Figure 4G, H, K, L)

**Figure 4:** Comparative immunohistochemical analysis with antibodies against full length or calpain-cleaved a-syn in passively immunized a-syn tg mice. To examine the effects of immunization on α-syn accumulation, immunohistochemical analysis using antibodies against FL-α-syn (layers 5–6) and CC-α-syn was conducted. Panels illustrate laser scanning confocal images of the temporal cortex and hippocampus (CA3) immunolabeled with antibodies against FL and CC α-syn immunoreactivity. (A, C) Temporal cortex of IgG1-immunized non-tg and α-syn tg mouse immunolabeled with an antibody against FL-α-syn, respectively. (B, D) Temporal cortex of 9E4-immunized non-tg and α-syn tg mouse immunolabeled with an antibody against FL-α-syn, respectively. (E, G) Hippocampus of IgG1-immunized non-tg and α-syn tg mouse immunolabeled with an antibody against FL-α-syn, respectively. (F, H) Hippocampus of 9E4-immunized non-tg and α-syn tg mouse immunolabeled with an antibody against FL-α-syn, respectively. (I) Image analysis of the numbers of neocortical α-syn immunoreactivity neurons with the FL α-syn antibody. (J) Analysis of the levels of α-syn immunoreactivity in the neuropil in the neocortex in sections labeled with the FL α-syn antibody. (K) Image analysis of the numbers of hippocampal α-syn immunoreactivity neurons with the FL α-syn antibody. (L) Analysis of the levels of α-syn immunoreactivity in the neuropil in the hippocampus in sections labeled with the FL α-syn antibody. (M, O) Temporal cortex of IgG1-immunized non-tg and α-syn tg mouse immunolabeled with an antibody against CC α-syn, respectively. (N, P) Temporal cortex of 9E4-immunized non-tg and α-syn tg mouse immunolabeled with an antibody against CC α-syn, respectively. (Q, S) Hippocampus of IgG1-immunized non-tg and α-syn tg mouse immunolabeled with an antibody against CC α-syn, respectively. (R, T) Hippocampus of 9E4-immunized non-tg and α-syn tg mouse immunolabeled with an antibody against CC α-syn, respectively. (U) Image analysis of the numbers of neocortical α-syn immunoreactivity neurons with the CC α-syn antibody. (V) Analysis of the levels of α-syn immunoreactivity in the neuropil in the neocortex in sections labeled with the CC α-syn antibody. (W) Image analysis of the numbers of hippocampal α-syn immunoreactivity neurons with the CC α-syn antibody. (X) Analysis of the levels of α-syn immunoreactivity in the neuropil in the hippocampus in sections labeled with the CC α-syn antibody. Scale bar  = 30 µM. N = 20 mice per group; 12 month old. Error bars represent mean ± SEM. (*) indicates p<0.05, when comparing IgG1-immunized α-syn tg mice to IgG1-imunized non-tg mice by one-way ANOVA with post hoc Dunnett's. (#) Indicates p<0.05, when comparing α-syn tg mice immunized the 9E4 α-syn antibody to IgG1-treated α-syn tg mice by one-way ANOVA with post hoc Dunnett's.

In contrast, immunohistochemical analysis with the antibody against CC α-syn showed a significant reduction in the levels of immunoreactivity in the both the numbers of immunolabeled intra-neuronal aggregates and the neuropil in the temporal cortex and hippocampus in the α-syn tg mice treated with the 9E4 antibody when compared to α-syn tg mice treated with the IgG1 control (temporal cortex, Figure 4O, P, U, V), hippocampus, Figure 4S, T, W, X).

In the temporal cortex of α-syn tg mice immunized with the 9E4 antibody intra-neuronal α-syn immunoreactivity, as detected by the CC-α-syn antibody was reduced 43% when compared to α-syn tg mice treated with the IgG1 control. Similarly, neocortical α-syn immunoreactive neuropil in α-syn tg mice immunized with the 9E4 antibody displayed a 57% reduction in the accumulation of CC α-syn when compared to α-syn tg mice treated with the IgG1 control. In the hippocampus of α-syn tg mice immunized with the 9E4 antibody intra-neuronal α-syn immunoreactivity, as detected by the CC-α-syn antibody was reduced 90% when compared to α-syn tg mice treated with the IgG1 control.

Hippocampal α-syn immunoreactive neuropil in α-syn tg mice immunized with the 9E4 antibody displayed a 33% reduction in the accumulation of CC α-syn when compared to α-syn tg mice treated with the IgG1 control.

In the IgG1- or 9E4-treated non-tg mice the FL and CC-α-syn antibodies detected minimal levels of α-syn in neocortical or hippocampal neurons (Figure 4A, B, I, E, F, K, M, N, U, V, Q, R, W, X). However the FL α-syn antibody was able to detect low levels of α-syn in the neuropil of these regions in the non-tg mice (Figure 4A, J, E, L).

Consistent with immunohistochemical findings, immunoblot analysis with the polyclonal antibody against FL α-syn (Figure 5A) showed similar levels of α-syn monomer (Figure 5B) and oligomer species (Figure 5C) in the soluble fraction of 9E4-treated α-syn tg mice when compared IgG1-treated α-syn tg mice. Levels of α-syn oligomers in the insoluble fraction were significantly reduced in the α-syn tg mice immunized with the 9E4 antibody compared to IgG1-treated α-syn tg mice (Figure 5D, F), whilst levels of α-syn monomers were low and appeared unaffected by immunization (Figure 5D, E).

**Figure 5:** Immunoblot analysis with antibodies against full length and calpain-cleaved a-syn in passively immunized α-syn tg mice. To evaluate the effects of immunization on α-syn accumulation, immunoblot analysis using antibodies against FL-αsyn and CC-α-syn was conducted. (A) Representative immunoblot with anti-FL α-syn of the soluble fraction from non-tg and α-syn tg mice immunized with IgG1 control or 9E4. (B, C) Analysis of the levels of the α-syn immunoreactive bands corresponding to the monomer and oligomers respectively, as detected by the FL α-syn antibody in the soluble fraction. (D) Representative immunoblot with anti-FL α-syn of the insoluble fraction from non-tg and α-syn tg mice immunized with IgG1 control or 9E4. (E, F) Analysis of α-syn monomer or oligomer levels respectively, detected by the FL α-syn antibody in the insoluble fraction. (G) Representative immunoblot with anti-CC α-syn of the soluble fraction from non-tg and α-syn tg mice immunized with IgG1 control or 9E4. (H, I) Analysis of α-syn monomer or oligomer levels respectively detected by the CC α-syn antibody in the soluble fraction. (J) Representative immunoblot with anti-CC α-syn of the insoluble fraction from non-tg and α-syn tg mice immunized with IgG1 control or 9E4. (K, L) Analysis of α-syn monomer or oligomer levels respectively, detected by the CC α-syn antibody in the insoluble fraction. N = 20 mice per group; 12 month old. Error bars represent mean ± SEM. (*) indicates p<0.05, when comparing IgG1-immiunized α-syn tg mice with IgG1-immunized non-tg mice using one-way ANOVA with post hoc Dunnett's. (#) indicates p<0.05, when comparing α-syn tg mice immunized with 9E4 with IgG1 immunized α-syn tg mice using one-way ANOVA with post hoc Dunnett's.

Immunoblot analysis with the antibody against CC α-syn in the soluble fraction showed a significant decrease in α-syn monomers and oligomers in 9E4-treated α-syn tg mice, in comparison to the IgG1-treated α-syn tg mice (Figure 5G–I). In the insoluble fraction the CC α-syn antibody showed a reduction of approximately 70% in the levels of monomeric α-syn band (Figure 5J, K) and a 95% reduction in the levels of the bands corresponding to oligomers in the insoluble fraction in the 9E4-treated α-syn tg mice group in comparison to the IgG1-treated α-syn tg mice (Figure 5J, L). In the non-tg mice immunization with the 9E4 antibody had no effect upon levels of FL- or CC-α-syn (Figure 5).

Given the recent results from genome-wide association studies suggesting that tau may play an important role in α-synucleinopathies such as PD [39], [40] we examined the effect of passive immunization with 9E4 on levels of tau and PHF-tau in the α-syn tg mice (Figure S2). Immunohistochemical analysis of the frontal cortex using an antibody against tau did not show significantly different levels of total tau between IgG1-treated α-syn tg and non-tg mice (Figure S2A, C, E), in contrast, IgG1-treated α-syn tg mice had significantly higher levels of PHF-tau, a four-fold increase in comparison to IgG1-treated non-tg mice (Figure S2F, H, J). 9E4 immunization did not alter levels of total tau (Figure S2B, D, E,) or PHF-tau (Figure S2G, I, J) in either group. Immunoblot analysis of total and PHF-tau levels was consistent with the immunohistochemical results and demonstrated no effect of 9E4 immunization on levels of total or PHF-tau in α-syn tg or non-tg mice (Figure S2K–M).

As passive immunization has been suggested to perturb vasculature we performed immunohistochemical analysis with the endothelial cell marker Zo-1 to examine the effects of immunization with the 9E4 antibody. In IgG1-treated non-tg and α-syn tg mice Zo-1 immunoreactivity was observed in the neuropil in association with the microvasculature and immunization with 9E4 had no effect upon Zo-1 immunoreactivity in either group (Figure S3A–E).

Immunohistochemical analysis of glial cell reactivity surrounding the vasculature was performed using markers against microglial and astroglial activation (Iba-1 and GFAP, respectively). IgG1- and 9E4-treated non-tg mice showed similar patterns of Iba-1 immunoreactivity in the neuropil around the blood vessels (Figure S3F, G, J). There was a moderate increase in Iba-1 immunoreactive microglial cells in the IgG1-treated α-syn tg mice in comparison to the IgG1-treated non-tg mice (Figure S3F, H, J) and no difference in Iba-1 immunoreactivity was observed the IgG1- or 9E4-treated α-syn tg mice (Figure S3H–J).

In the non-tg mice scattered GFAP immunoreactive astroglial cells were observed in the neuropil surrounding blood vessels (Figure S3K), no differences in the levels of GFAP were observed between IgG1- and 9E4-treated non-tg mice (Figure S3K, L, O). In contrast, the IgG1-treated α-syn tg mice had a robust increase in GFAP immunoreactivity in comparison to the IgG1-treated non-tg mice (Figure S3K, M, O) and passive immunization with 9E4 was able to reduce GFAP immunoreactivity in the α-syn tg mice (Figure S3M–O) resulting in a normalization of astroglial cells around the blood vessels in these mice.

Collectively the results thus far demonstrate that the 9E4 antibody is specific for human α-syn, significantly ameliorates the motor and memory/learning deficits examined in the α-syn tg mice and is effective at reducing the accumulation of α-syn in α-syn tg mice. Additionally these beneficial effects of 9E4 did not perturb the microvasculature.

### A monoclonal antibody against CT-α-syn traffics into the CNS and localizes to lysosomes

In order to evaluate the trafficking of 9E4 into the CNS, 9E4 and a control IgG1 were labeled with FITC and injected intravenously into non-tg and α-syn tg. At 3 days post injection low levels of the 9E4 antibody were detected in the brain, while high levels were detected in plasma (Figure 6A). At 14 and 30 days post injection higher levels were detected in the brain with decreasing levels in the plasma as detected by ELISA (Figure 6A). By immunohistochemistry the 9E4-FITC antibody was detected in association with neurons in the brains of α-syn tg mice at 30 days post injection (Figure 6B). The 9E4-FITC antibody was detected in association with granular structures in neurons distributed in the deeper layers of the temporal cortex and the CA1-2 region of the hippocampus only in the brains of α-syn tg mice (Figure 6C, D). Control experiments with a non-immune IgG1-FITC show only background labeling in α-syn tg mice (Figure 6E). In non-tg mice only low levels of 9E4-FITC labeling were detected in blood vessels (Figure 6F).

**Figure 6:** Trafficking of the FITC-tagged α-syn 9E4 antibody in tg mice. To investigate the distribution of the 9E4 antibody after passive immunization, the FITC tagged antibody was injected intravenously (IV) and analyzed by ELISA and confocal microscopy. (A) Antibody titers in the plasma and brain at 3, 14 and 30 days post-injection in mice immunized with the 9E4 antibody, determined by ELISA. (B) Image analysis of 9E4-FITC positive neurons in the α-syn tg mice at 3, 14 and 30 days post-injection. (C, D) Representative laser scanning confocal images of the signal in the FITC channel in the temporal cortex of α-syn tg mouse 30 days following intravenous IV injection with the FITC-tagged 9E4 antibody. Arrows highlight labeled intra-neuronal granular-like structures. (E) No signal is detected in the FITC channel in α-syn tg mouse 30 days following IV injection with the FITC-tagged IgG1 control antibody. (F) No signal in the FITC channel in non-tg mouse 30 days following IV injection with the FITC-tagged 9E4 antibody. (G) Confocal image of a section from an antibody-naive α-syn tg mouse immunolabeled with cerebrospinal fluid (CSF) from a mouse immunized with 9E4-FITC. (H) Confocal image of a section from non-tg mouse immunolabeled 9E4-FITC antibody. Scale bar (C, E–H)  = 50 µM; (D)  = 10 µM. N = 20 per group, 12 months of age. Error bars represent mean ± SEM.

To further confirm that the 9E4-FITC antibody crossed the blood-brain barrier (BBB) and circulated in the CNS, CSF from mice immunized with the IgG-FITC or 9E4-FITC antibodies was used to label sections from antibody-naive α-syn tg mice. These studies demonstrated that the CSF from mice immunized with the 9E4-FITC antibody immunolabeled synapses and neurons in the antibody-naive α-syn tg (Figure 6G), in contrast no labeling was observed with the CSF of mice treated with non-immune IgG1-FITC (Figure 6H).

As an additional control to assess the passage of a FITC-labeled protein into the brain, α-syn tg and non-tg mice were injected with FITC-labeled β-syn (Figure S4). No signal in the FITC channel was observed upon direct visualization of cortical sections from these mice (Figure S4A, B), as would be expected given that β-syn is a predominantly cytoplasmic protein and, unlike α-syn, has not been reported at the plasma membrane. However when CSF from mice injected with the FITC-labeled β-syn was used to immunolabel sections from naive α-syn tg and non-tg mice (those that had not been injected with the FITC-β-syn), a clear immunoreactivity was observed in the cortex of both non-tg and α-syn tg mice (Figure S4C and D).

To determine whether α-syn co-localizes to the structures decorated by 9E4-FITC, co-labeling experiments were performed. Laser scanning confocal microscopy in sections from α-syn tg mice showed that the granular structures within the neurons labeled with 9E4-FITC antibody co-localized with α-syn immunoreactivity (Figure 7A–C). These, intra-neuronal structures labeled by the 9E4-FITC displayed LC3 (Figure 7D–F) and cathepsin-D immunoreactivity (Figure 7G–I). To corroborate the localization of the 9E4 antibody to the lysosomes, immuno-electron microscopic analysis was performed with a gold-tagged anti-mouse antibody. Ultrastructural analysis confirmed the presence of immunogold particles in the lysosomes and autophagosomes in the brains of α-syn tg mice treated with 9E4 (Figure 7J, K). In contrast, no specific labeling of lysosomes or autophagosomes was detected in the brains of α-syn tg mice treated with the non-immune IgG1 (Figure 7L, M) or in the neurons non-tg mice treated with 9E4 (Figure 7N, O).

**Figure 7:** Co-localization of the FITC-tagged α-syn 9E4 antibody with lysosomal and autophagosomal markers. To analyze the sub-cellular distribution of the 9E4 antibody immunohistochemical and ultrastructural analysis was conducted in 9E4-FITC immunized α-syn tg mice. (A–C) Representative confocal image of a brain section from an α-syn tg mouse immunized 9E4-FITC and co-labeled with an antibody against α-syn. Arrows indicate co-localization of the 9E4-FITC signal with α-syn in neuronal granular-like structures. (D–F) Confocal image from an α-syn tg mouse immunized 9E4-FITC and co-labeled with an antibody against LC3. Arrows indicate co-localization of the 9E4-FITC with LC3 in neuronal autophagosome-like structures. (G–I) Confocal image from an α-syn tg mouse immunized 9E4-FITC and co-labeled with an antibody against cathepsin D. Arrows indicate co-localization of the 9E4-FITC with cathepsin-D in neuronal lysosomal-like structuresLC3. (J, K) Representative electron micrographs of sections from an α-syn tg mouse immunized with the 9E4 antibody and immunolabeld with gold-tagged anti-mouse antibody. (L, M) Electron micrographs of sections from an α-syn tg mouse immunized with the control IgG1 antibody and immunolabeld with gold-tagged anti-mouse antibody. (N, O) Representative electron micrographs of sections from a non-tg mouse immunized with the 9E4 antibody and immunolabeld with gold-tagged anti-mouse antibody. No reactivity is observed in lysosomes or autophagosomes. Scale bar (A–I)  = 10 µM; (J–O) magnification 25,000x.

Taken together, these studies suggest that the 9E4 antibody can cross the BBB and bind α-syn and it is possible that the resulting antibody-antigen complex may then be endocytosed and transferred into the lysosomal compartment for degradation.

### Passive immunotherapy with a monoclonal antibody against CT-α-syn activates the autophagy pathway

Since passive immunotherapy in this system appears to promote clearance of α-syn via a lysosomal pathway we investigated whether treatment with the 9E4 antibody activated the autophagy pathway in the α-syn tg immunized mice. Compared to control experiments where α-syn tg mice treated with IgG1 displayed discrete LC3 and cathepsin-D immunoreactivity granules, in the α-syn tg mice treated with the 9E4 antibody there was a significant increase in the neuronal levels of LC3 (Figure 8A-C) and cathepsin-D immunoreactivity (Figure 8D–F) This was accompanied by a decrease in the levels of intra-neuronal and synaptic CC α-syn accumulation and the compartmentalization of α-syn to granular structures (Figure 8G-I). Double labeling experiments confirmed that in the α-syn tg mice treated with the 9E4 antibody α-syn colocalized with the lysosomal (cathepsin-D) (Figure 8J–L) and autophagy (LC3) (Figure 8M–O) markers. Additional immunohistochemical was performed to confirm the co-localization of α-syn with LC3 in the 9E4 treated α-syn tg mice, which was absent in the IgG1 controls (Figure S5A–I). Further electron microscopy demonstrated a significant increase in the levels of gold-labeled α-syn particles in the phagosomes of 9E4 immunized α-syn tg mice in comparison to IgG1 controls (Figure S5J–N). Consistent with the immunohistochemistry, immunoblot analysis showed levels of LC3 breakdown and Beclin-1 immunoreactivity were increased in α-syn tg mice treated with the 9E4 antibody compared to the non-immune IgG1 (Figure 9A, B). Other genes expressed during autophagy, such as Atg 7 and Atg 10, remained stable with the 9E4 treatment in the α-syn tg mice (Figure 9A, B).

**Figure 8:** Immunocytochemical analysis of the effects of passive immunization with 9E4 in markers of lysosomes and autophagy in α-syn tg mice. To examine the sub-cellular distribution of the 9E4 antibody immunohistochemical and ultrastructural analysis was conducted in 9E4 immunized α-syn tg mice. (A) LC3 immunoreactivity in α-syn tg mouse immunized with IgG1 antibody. (B) LC3 immunoreactivity in α-syn tg mouse immunized with 9E4 antibody. (C) Analysis of LC3 immunoreactivity in α-syn tg mice immunized with IgG1 or 9E4 antibody. (D) Cathepsin-D immunoreactivity in α-syn tg mouse immunized with IgG1 antibody. (E) Cathepsin-D immunoreactivity in α-syn tg mouse immunized with 9E4 antibody. (F) Analysis of cathepsin-D immunoreactivity in α-syn tg mice immunized with IgG1 or 9E4 antibody. (G) CC α-syn immunoreactivity in α-syn tg mouse immunized with IgG1 antibody. (H) CC α-syn immunoreactivity in α-syn tg mouse immunized with 9E4 antibody. (I) Analysis of % area of CC α-syn immunoreactive neuropil in α-syn tg mice immunized with IgG1 or 9E4 antibody. (J–L) Co-localization of α-syn and cathepsin-D immunoreactivity in α-syn tg mouse immunized with 9E4 antibody. (M–O) Co-localization of α-syn and LC3 immunoreactivity in α-syn tg mouse immunized with 9E4 antibody. Scale bar (A, B)  = 30 µM (D, E, G and H)  = 20 µM, (J–O)  = 10 µM. (*) Indicates p<0.05, when comparing IgG1 to 9E4 group by unpaired Student's t test. Error bars represent mean ± SEM.

**Figure 9:** Immunoblot analysis of the effects of passive immunization with 9E4 in molecular components of the autophagy pathway in α-syn tg mice. (A) Immunoblot analysis of mTor, Beclin 1, LC3, Atg 5, Atg 7, and Atg 10 protein immunoreactivity in α-syn tg mice that had been immunized with either the IgG1 control or 9E4 antibody. (B) Analysis of mTor, Beclin 1, LC3, Atg 5, Atg 7, and Atg 10 protein levels in α-syn tg mice that had been immunized with either the IgG1 control or 9E4 antibody. (*) Indicates p<0.05, when comparing IgG1 to 9E4 group by unpaired Student's t test. Error bars represent mean ± SEM.

To confirm that the 9E4 antibody promotes clearance of α-syn aggregates via autophagy, *in vitro* experiments were performed in a neuronal cell line (B103 rat neuroblastoma cells [34]) expressing Lenti-virus (LV) α-syn and the reporter gene LC3-GFP. Under basal conditions neuronal cells expressing a control LV and treated with IgG1 only displayed discrete LC3-GFP granules (Figure 10A). Neuronal cells overexpressing α-syn showed the presence of enlarged LC3-GFP granules that co-localized with a-syn (Figure 10B). Treatment of the neuronal cells infected with the LV- α-syn with the 9E4 antibody resulted in an increase number of normal appearing LC3-GFP granules with a considerable decrease in the accumulation of α-syn in the cytoplasm (Figure 10C). In these neuronal cells, granular α-syn deposits co-localized to LC3-GFP structures representing autophagosomes (Figure 10C). The effects of the 9E4 antibody at reducing α-syn and elevating LC3-GFP were enhanced by rapamycin (an inducer of autophagy) (Figure 10E, G and H) and were blocked by 3-MA (an inhibitor of autophagy) (Figure 10F, I and J).

**Figure 10:** The effects of the 9E4 monoclonal antibody on promotion of α-syn clearance via autophagy in a neuronal cell model. (A) Baseline co-localization of α-syn and LC3-GFP in neuronal cells infected with LV-control and treated with the IgG1 control antibody. (B) Baseline co-localization of α-syn and LC3-GFP in neuronal cells infected with LV-α-syn and treated with the IgG1 control antibody. (C) Co-localization of α-syn and LC3-GFP in neuronal cells infected with LV-α-syn and treated with the 9E4 antibody. (D) Co-localization of α-syn and LC3-GFP in neuronal cells infected with LV-control, treated with the IgG1 control antibody and rapamycin, an inducer of autophagy. (E) Co-localization of α-syn and LC3-GFP in neuronal cells infected with LV-α-syn, treated with the 9E4 antibody and rapamycin, an inducer of autophagy. (F) Co-localization of α-syn and LC3-GFP in neuronal cells infected with LV-α-syn, treated with the 9E4 antibody and 3MA, an inhibitor of autophagy. (G) Analysis of α-syn immunoreactivity in neuronal cells infected with LV-α-syn, treated with the 9E4 antibody and rapamycin. (H) Analysis of LC3-GFP signal in neuronal cells infected with LV-α-syn, treated with the 9E4 antibody and rapamycin. (I) Analysis of α-syn immunoreactivity in neuronal cells infected with LV-α-syn, treated with the 9E4 antibody and 3MA. (J) Quantitative analysis of LC3-GFP signal in neuronal cells infected with LV-α-syn, treated with the 9E4 antibody and 3MA. Scale bar (A–F)  = 10 µM (*) Indicates p<0.05 compared to LV-control infected and vehicle-treated cultures by one-way ANOVA with post-hoc Dunnett's test. (#) Indicates p<0.05 compared to LV-control infected and vehicle-treated cultures by one-way ANOVA with post-hoc Tukey-Kramer test. Error bars represent mean ± SEM.

Taken together, these results support the possibility that passive immunization with antibodies against the CT of α-syn promotes clearance of α-syn aggregates via autophagy.

## Discussion

The present study is the first to demonstrate that passive immunization with an antibody directed at the CT of α-syn is able to reduce memory/learning deficits and promote clearance of cortical and hippocampal a-syn aggregates in tg mice expressing human α-syn under the PDGFβ promoter. This is consistent with a previous study utilizing active immunization where epitope mapping indicated that the best results in terms of reducing a-syn was observed with antibodies that preferentially recognize the CT of a-syn [17]. Though the reason for the enhanced activity of the antibodies against the CT of a-syn is not completely understood, recent studies have supported the possibility that the generation of neurotoxic a-syn aggregates involves CT cleavage [41] and interactions with the CT domain of a-syn [10], [42]. Therefore it is possible that antibody targeting of this region may reduce the generation of this toxic species.

Calcium dependent calpain activation cleaves a-syn at the CT between amino acids 121–123 [32]. The cleavage of a-syn at either the NT or CT end of a-syn could be detected in the brains of patients with PD and DLB using two site-directed calpain-cleavage antibodies [32]. Calpain can cleave a-syn in vitro, leading to its aggregation and adoption of a b-sheet conformation. Therefore, immunization with antibodies against the CT of a-syn might be protective either by blocking the CT cleavage of a-syn, recognizing and promoting the clearance of CT fragments and aggregates of a-syn or by blocking the interaction of CT fragments with FL a-syn. In support of this possibility the present study showed that passive immunotherapy reduced the accumulation and formation of CT fragments compared to FL a-syn. The antibody against the calpain-cleaved a-syn utilized for this study has been shown to recognize both the free a-syn fragments as well as those complexed in oligomers [32]. These antibodies are sensitive at recognizing sets of a-syn aggregates that appear relevant to the disease process, given that such immunoreactivity is not found in control cases or other neurodegenerative disorders [32], [43]. In the brains of patients with DLB as well as in the tg models, a-syn aggregates containing CT-fragments not only accumulate in the cell bodies but also in axons and nerve terminals. In the tg animals, immunotherapy reduced the accumulation of a-syn preferentially in the neuropil. This was associated with improved behavioral performance in the water maze and expression of the post-synaptic markers such as PSD95. This is consistent with recent studies supporting the view that neurotoxic a-syn accumulates preferentially in synapses and that a-syn interferes with synaptic function [44], [45]. Therefore promoting the clearance of a-syn aggregates could be beneficial and result in functional improvements.

Potential explanations for the preferential beneficial effects of antibodies against the CT of a-syn include the possibility the CT epitopes in a-syn might be more readily exposed facilitating recognition by the antibody. For example, molecular modeling and nuclear magnetic resonance studies suggest that while the NT of a-syn interacts with the membrane [22], the CT tail is more rigid [46], capable of penetrating the membrane and be freely exposed to the external membrane surface where it can be recognized by the antibodies [21], [22]. Given that under physiological conditions a-syn is primarily a cytosolic protein it is puzzling how the antibodies utilized for the passive immunization strategies described in this study might recognize and trigger the clearance of a-syn. In this regard it is worth noting that under pathological condition the aggregated a-syn tends to accumulate in the membrane [21], [47], [48], [49] and to be exposed to the extracellular compartment. Moreover, neurotoxic a-syn oligomers can be secreted via exosomes into the extracellular space [50], [51], [52] and can be detected in the CSF [26], [53]. This suggests that the antibodies might recognize a-syn aggregates lying in the cell surface that in turn might be internalized and cleared via the autophagy pathway. In support of this possibility, in the present study we showed that systemically administered FITC-tagged antibodies against a-syn traffic into the CNS and are internalized by a-syn containing neurons and identified by double labeling and immunogold in lysosomes and autophagosomes. Moreover, a-syn was detected in LC3-positive granular structures further supporting a role for the autophagy-mediated clearance of a-syn in the immunized animals. This is consistent with recent studies showing that activating the autophagy pathway with pharmacological [54], [55] or gene therapy approaches promote elimination of a-syn aggregates and ameliorates the deficits in tg mice [12], [15].

Previous work by our group has shown that active immunization with recombinant α-syn ameliorates α-syn related synaptic pathology in a tg mouse model of PD [17], however given the common immunological problems that have often been associated with active immunization we chose to pursue a passive immunization protocol for this study. Our results indicate that passive immunization is as effective as active for the sequestration and removal of α-syn aggregates. It is interesting to note that both the passive and active immunization approaches to α-syn eventually result in the recruitment of the autophagocytic pathway indicating that key mechanisms may be involved in the degradation of α-syn.

Passive immunization with antibodies against amyloid-beta (Ab has been extensively investigated as a potential treatment modality for AD [56], [57], [58], [59]. These studies have been bolstered by the fact that Ab is secreted and easily accessible to antibody recognition. However a number of recent studies have shown that similarly to a-syn, immunotherapy can reduce the accumulation of other membrane bound and intracellular protein aggregates such as tau [60], [61], PrP [62] and huntingtin [63].

In conclusion, we show that a monoclonal antibody against CT α-syn traffics into the CNS, recognizes α-syn aggregates in affected neurons and ameliorates behavioral and neuropathological alterations in α-syn tg mice. Taken together, the results from this study support the view that passive immunization with antibodies against the CT of a-syn might have therapeutic potential in the treatment of PD and DLB.

## Supporting Information

Figure S1 **Immunochemical characterization of the specificity of a-syn antibodies utilized for passive immunotherapy.** Immunoblot and immunohistochemical analysis was conducted to characterize the different α-syn antibodies and to select the one that was subsequently used for passive immunotherapy. Western blot analysis was performed with soluble fraction from the temporal cortex. (A) Immunoblot analysis in non-tg and α-syn tg mice with IgG1 control and the mouse monoclonal antibodies against -α-syn- 6H7, 8A5, 9E4 and the polyclonal antibodies against full-length (FL) α-syn and Calpain cleaved (CC) α-syn. (B, C) Background levels of immunostaining with the control IgG1 in non-tg and α-syn tg, respectively. (D, E) Representative confocal images with the 6H7 antibody in non-tg and α-syn tg, displaying immunostaining in the neuropil and neurons in the temporal cortex respectively. (F, G) Confocal images with the 8A5 antibody in non-tg and α-syn tg, displaying immunostaining in the neuropil and neurons respectively. (H, I) Confocal images with the 9E4 antibody in non-tg showing no specific labeling and immunostaining in the neuropil and neurons in α-syn tg. (J, K) FL α-syn immunoreactivity in non-tg and α-syn tg, respectively. (L, M) CC α-syn immunoreactivity in non-tg and α-syn tg, respectively). N =  3 per group, 6 months of age. Scale bar (B-M)  =  30μM.
(TIF)

Figure S2 **Effects of passive immunization with a C-terminal α-syn antibody on tau.** Levels of total and PHF-tau were examined by immunohistochemistry and immunoblot analysis to asses the effects of passive immunization with 9E4. (A, B) Representative brightfield images of total tau in the frontal cortex of IgG1- and 9E4-treated non-tg mice, respectively. (C, D) Representative brightfield images of total tau in the frontal cortex of IgG1- and 9E4-treated α-syn tg mice, respectively. (E) Quantitative analysis of total tau levels in the frontal cortex of IgG1 and 9E4-treated non-tg and α-syn tg mice. (F, G) Representative brightfield images of PHF-tau in the frontal cortex of IgG1- and 9E4-treated non-tg mice, respectively. (H, I) Representative brightfield images of PHF-tau in the frontal cortex of IgG1- and 9E4-treated α-syn tg mice, respectively. (J) Quantitative analysis of PHF-tau levels in the frontal cortex of IgG1 and 9E4-treated non-tg and α-syn tg mice. (K) Immunoblot of levels of total and PHF-tau in the frontal cortex of IgG1 and 9E4 treated non-tg and α-syn tg mice. (L) Analysis of total tau levels in the frontal cortex of IgG1 and 9E4-treated non-tg and α-syn tg mice as determined by immunoblot. (M) Analysis of PHF-tau levels in the frontal cortex of IgG1 and 9E4-treated non-tg and α-syn tg mice as determined by immunoblot. Scale bar  =  40uM. Error bars represent mean ± SEM. (*) Indicates p<0.05, when comparing α-syn tg immunized with IgG1 or 9E4 to IgG1-treated non-tg mice by one-way ANOVA with post hoc Dunnett's.
(TIF)

Figure S3 **Effects of passive immunization with a C-terminal α-syn antibody on vasculature or markers of glial cell reactivity.** (A, B) Representative brightfield images of the endothelial cells marker Zo-1 immunoreactivity in the frontal cortex of IgG1- and 9E4-treated non-tg mice, respectively (arrows indicate location of blood vessels). (C, D) Representative brightfield images of Zo-1 immunoreactivity in the frontal cortex of IgG1- and 9E4-treated α-syn tg mice, respectively (arrows indicate location of blood vessels). (E) Analysis of % of Zo-1 immunoreactive neuropil in the frontal cortex of IgG1- and 9E4-treated non-tg and α-syn tg mice. (F, G) Representative brightfield images of the microglial marker Iba-1 immunoreactivity in the frontal cortex of IgG1- and 9E4-treated non-tg mice, respectively. (G, H) Representative brightfield images of Iba-1 immunoreactivity in the frontal cortex of IgG1- and 9E4-treated α-syn tg mice, respectively. (E) Analysis of Iba-1 immunoreactivity in the frontal cortex of IgG1- and 9E4-treated non-tg and α-syn tg mice. (F, G) Representative brightfield images of the microglial marker Iba-1 immunoreactivity in the frontal cortex of IgG1- and 9E4-treated non-tg mice, respectively. (K, L) Representative brightfield images of the astroglial cell marker GFAP immunoreactivity in the frontal cortex of IgG1- and 9E4-treated non-tg mice, respectively (arrows indicate location of blood vessels). (M, N) Representative brightfield images of GFAP immunoreactivity in the frontal cortex of IgG1- and 9E4-treated α-syn tg mice, respectively (arrows indicate location of blood vessels). (E) Analysis of GFAP immunoreactivity in the frontal cortex of IgG1- and 9E4-treated non-tg and α-syn tg mice. Scale bar (A-D)  =  80uM, (F-N)  =  50μM. Error bars represent mean ± SEM. (*) indicates p<0.05, when comparing IgG1-immunized α-syn tg mice to IgG1-imunized non-tg mice by one-way ANOVA with post hoc Dunnett's. (#) Indicates p<0.05, when comparing α-syn tg mice immunized the 9E4 α-syn antibody to IgG1-treated α-syn tg mice by one-way ANOVA with post hoc Dunnett's.
(TIF)

Figure S4 **FITC-labeled β-syn crosses the blood-brain barrier but does not bind neurons in α-syn tg mice.** (A, B) Signal in the FITC channel upon direct visualization of temporal cortex sections from non-tg and α-syn tg mice injected with FITC-labeled β-syn, respectively. (C, D) Representative confocal images of the neocortex of non-tg and α-syn mice, respectively, immunolabeled with CSF from mice injected with FITC-labeled β-syn displaying immunostaining of the neuropil. Scale bar (A-I)  =  10μM.
(TIF)

Figure S5 **Further characterization of LC3 immunoreactivity and phagosome involvement of α-syn clearance in α-syn tg mice immunized with 9E4.** (A) α-syn immunoreactivity in α-syn tg mouse immunized with the IgG1 control antibody. (B) LC3 immunoreactivity in α-syn tg mouse immunized with the IgG1 control antibody. (C) Co-localization of α-syn and LC3 immunoreactivity in α-syn tg mouse immunized with the IgG1 control antibody. (D, G) α-syn immunoreactivity in α-syn tg mouse immunized with the 9E4 antibody. (E, H) LC3 immunoreactivity in α-syn tg mouse immunized with the 9E4 antibody. (F, I) Co-localization of α-syn and LC3 immunoreactivity in α-syn tg mouse immunized with the 9E4 antibody. (J, K) Immuno-gold electron micrographs of phagosomes from α-syn tg mouse immunized with the IgG1 control antibody, very few gold particles were detected. (L, M) Immuno-gold electron microscopy images of phagosomes from α-syn tg mouse immunized with the 9E4 antibody, abundant gold particles were detected.(N) Quantitative analysis of gold particles in phagosomes from α-syn tg mice immunized with either IgG1 control or 9E4 antibody Scale bar (A-I)  =  10μM (J-M)  =  0.5μM Error bars represent mean ± SEM. (*) Indicates p<0.05, when comparing IgG1 to 9E4 group by one way ANOVA with post hoc Dunnet's.
(TIF)
